# Fusion-Based Deep Learning with Nature-Inspired Algorithm for Intracerebral Haemorrhage Diagnosis

**DOI:** 10.1155/2022/4409336

**Published:** 2022-01-18

**Authors:** Nada M. Alfaer, Hassan M. Aljohani, Sayed. Abdel-Khalek, Abdulaziz S. Alghamdi, Romany F. Mansour

**Affiliations:** ^1^Department of Mathematics and Statistics, College of Science, Taif University, Taif 21944, Saudi Arabia; ^2^Department of Mathematics, Sohag University, Sohag 82524, Egypt; ^3^Department of Mathematics, College of Science and Arts, King Abdulaziz University, P. O. Box 344, Rabigh 21911, Saudi Arabia; ^4^Department of Mathematics, New Valley University, El-Kharga 72511, Egypt

## Abstract

Natural computing refers to computational processes observed in nature and human-designed computing inspired by nature. In recent times, data fusion in the healthcare sector becomes a challenging issue, and it needs to be resolved. At the same time, intracerebral haemorrhage (ICH) is the injury of blood vessels on the brain cells, which is mainly liable for stroke. X-rays and computed tomography (CT) scans are widely applied for locating the haemorrhage position and size. Since manual segmentation of the CT scans by planimetry by the use of radiologists is a time-consuming process, deep learning (DL) is used to attain effective ICH diagnosis performance. This paper presents an automated intracerebral haemorrhage diagnosis using fusion-based deep learning with swarm intelligence (AICH-FDLSI) algorithm. The AICH-FDLSI model operates on four major stages namely preprocessing, image segmentation, feature extraction, and classification. To begin with, the input image is preprocessed using the median filtering (MF) technique to remove the noise present in the image. Next, the seagull optimization algorithm (SOA) with Otsu multilevel thresholding is employed for image segmentation. In addition, the fusion-based feature extraction model using the Capsule Network (CapsNet) and EfficientNet is applied to extract a useful set of features. Moreover, deer hunting optimization (DHO) algorithm is utilized for the hyperparameter optimization of the CapsNet and DenseNet models. Finally, a fuzzy support vector machine (FSVM) is applied as a classification technique to identify the different classes of ICH. A set of simulations takes place to determine the diagnostic performance of the AICH-FDLSI model using the benchmark intracranial haemorrhage data set. The experimental outcome stated that the AICH-FDLSI model has reached a proficient performance over the compared methods in a significant way.

## 1. Introduction

In the last few years, traumatic brain injury (TBI) is the primary cause of growing death rates and disability in the USA. Nearly 30% of injury deaths have been reported [1]. After that, TBI, extra-axial intracranial tumours such as intracranial hemorrhages (ICH), may take place. The ICH disease is the main reason for death worldwide that happens for all ages. At first, the disease is initiated in the brain due to the leakage in the blood vessel and removes the path of interactions (follows the brain function and instruction consequently) and internal organ that results in inactive body functions such as memory loss, loss of eyesight, speech, and so on [2–4]. The most important risk factors such as high blood pressure (BP), head trauma, leakage in veins, and infected blood vessel walls are related to the ICH. To inspect this disorder, the screening modalities such as single-photon emission computed tomography (SPECT), X-ray, positron emission tomography (PET), and computed tomography (CT) are accessed via brain haemorrhage imaging. In comparison to other methods, a CT scan is widely employed in haemorrhage diagnosis as it is widely available, limited duration, and inexpensive for imaging. Therefore, CT scans are highly desired for ICH detection. The manifestation of ICH clots on CT scans depends on external factors such as volume, density, location, and slice intensity.

The early prediction of ICH is indispensable for sufficient scheduling of scanning and providing better treatment. Therefore, enormous designers have used the computer-based detection (CAD) method for ICH segmentation. The recently proposed computer-based CAD method of ICH is based on the aspects such as automatic segmentation of haemorrhage that can be forecasted without manual segmentation, professional contribution, in which the human experts have to offer a suitable input for segmentation. The current deployment in convolutional neural network (CNN) and deep learning (DL) served remarkable performances in automatic image segmentation and classification processes [5]. Thus, the DL technique can able to make automated ICH segmentation and prediction.

In recent times, researchers have attempted to employ the DL technique for the diagnosis of ICH on CT scans [6]. This DL technique is a kind of machine learning (ML) that employs various processing layers to learn a representation of data with many levels of abstraction. Earlier researchers utilizing this technique presented tremendous diagnostic performances to detect ICH in every single CT scan, same as that of expert radiotherapists. Additionally, the fully 3D DL method (not on single CT scans) for diagnosing ICH has been stated. Few researchers utilized the back-propagation (BP) model for the learning approach and the CNN that has pattern recognition and self-organization capacities without human programming. Consequently, this method is a problem agnostic and generic technique, not a problem-specific and rule-based model [7]. But it remains challenging to explicate how this technique generates the outcomes from the input data.

This paper presents an automated intracerebral haemorrhage diagnosis using fusion-based deep learning with swarm intelligence (AICH-FDLSI) algorithm. The AICH-FDLSI model employs a seagull optimization algorithm (SOA) with Otsu multilevel thresholding is employed for image segmentation. Besides, the fusion-based feature extraction using the Capsule Network (CapsNet) and EfficientNet is applied to extract a useful set of features. At the same time, deer hunting optimization (DHO) algorithm is utilized for the hyperparameter optimization of the CapsNet and DenseNet models. Lastly, a fuzzy support vector machine (FSVM) is employed as a classifier to determine various classes of ICH. To showcase the improved classifier results of the proposed model, a wide range of experiments is performed using the test benchmark intracranial haemorrhage data set.

The rest of the study is planned as follows.  Section 2 provides the related works; Section 3 offers the proposed model; Section 4 discusses the performance validation; and Section 5 concludes the study.

## 2. Literature Review

Mansour et al. [8] proposed an innovative DL-based ICH diagnoses and classification (DL-ICH) method with the help of optimum image segmentation using inception network. The presented method includes segmentation, preprocessing, classification, and feature extraction. First, the input data undergoes conversion format in which the NIfTI files are transformed into JPEG form. Anupama et al. [9] presented DL-based ICH diagnoses with GrabCut-based segmentation using SDL, called GC-SDL algorithm. Furthermore, GrabCut-based segmentation is utilized to identify the infected portion efficiently in an image. To execute the process of feature extraction, the SDL method is employed, and lastly, the SM layer is applied as a classifier.

Venugopal et al. [10] proposed a unique multimodal data fusion-based feature extraction method using a DL algorithm, called FFE-DL for ICH Classification and Detection, named as FFEDL-ICH. The presented method consists of classification, preprocessing, image segmentation, and feature extraction. First, the input images are preprocessed by the GF method for removing noise. Next, the DFCM method is employed for segmenting the image. Moreover, the fusion-based feature extraction method is performed by deep features (residual network 152) and handcrafted features (local binary patterns) for extracting appropriate features. Lastly, the DNN method is performed as a classification method to distinguish different types of ICH. A new DL method for ANN, totally distinct from the BP algorithm, was proposed in earlier research [11]. The objective is to measure the possibility of utilizing the model for ICH classification and detection of its subclasses, without applying the CNN method.

Wang et al. [12] focused on evaluating the accuracy and performance of a DL-based automatic segmentation method in segmenting spontaneous ICH volume either with/without IVH extensions. They related this automatic method with two manual segmentation methods. Ginat [7] examines the execution of DL for the work list prioritization and detection of acute ICH on NCCT in different medical sceneries at an academic medical centre. The images were categorized based on the type and presence of haemorrhage, whether this is follow-up/initial images, and patient visit location, involving outpatient, emergency or trauma, and inpatient sections. Yu et al. [13] intended to improve a strong DL segmentation technique for accurate and fast HV analyses via CT. Luong et al. [14] presented a CAD that integrates a DL method and image processing methods for determining patient who suffers from ICH because of their CT scans. The DL method-based MobileNetV2 framework was trained.

Ngo et al. [15] developed a newfangled method for training slice-level classifier on CT-based descriptor of the nearby slices alongside the axis; all of them are extracted by the CNN method. This technique focuses on predicting the existence of ICH and categorizes it into five distinct subclasses. They examine a two-phase training system. Initially, CT images are processed simply as a group of two-dimensional images, and an advanced CNN classifier is trained that is pretrained on ImageNet. In the training phase, all the slices are tested together with the three slices beforehand and the three slices afterward, which makes the batch size a multiple of 7. Next, the output descriptor of all the blocks of seven successive slices attained from phase 1 are stacked into images and fed into other CNNs for the last predictions of middle slices. Hssayeni et al. [16] developed a method for collecting and eighty-two CT scan data sets of subjects with a traumatic brain injury. Then, the ICH regions were manually delineated in every slice by a consensus decision of two radiologists. The data set is an open-source platform at the PhysioNet repository for upcoming comparisons and analyses. Besides publishing the data set, that is, the major objective of this manuscript, they executed a deep FCN model called as UNet, for segmenting the ICH region from the CT images in a fully automatic methodology.

## 3. The Proposed Model

This paper has developed a novel AICH-FDLSI technique for ICH detection and classification. The proposed AICH-FDLSI technique encompasses MF-based preprocessing, SOA with Otsu multilevel thresholding-based segmentation, DHO-based feature extraction, and FSVM-based classification. The detailed working of these processes is offered in the succeeding sections.

### 3.1. Image Preprocessing

Primarily, the MF technique is applied as a preprocessing tool to eliminate the presence of noise involved in it. The MF is nonlinear statistical filtering that changes the existing pixel values with the median value of pixels under the adjacent area. A naive execution primary makes a cumulative histogram to the neighbor area and afterward defines the primary index elsewhere half the amount of pixels from the histograms. An essential issue of this manner on GPU is all the threads required for computing whole histograms. For 8-bit images, a histogram made of 256 bins is generated. It can be useless on present GP as there are not sufficient hardware registers obtainable to all the threads, and utilizing global memory to histogram calculation was too slow. For resolving this issue, the presented model depends upon a bisection search on histogram ranges. This technique does not calculate the actual histogram then iteratively improves the histogram range that contains the median value. In all rounds, the existing valid range was separated into two halves, and the half that is the huge amount of pixels is elected to the next iteration. This procedure was repeated still the range converged to a single bin.

### 3.2. Image Segmentation

During the image segmentation process, the SOA with Otsu multilevel thresholding is applied to determine the affected regions. The Otsu is also named as maximal difference between clusters [17]. An image histogram as fundamental and maximal difference between target as well as background as the selective condition, this technique obtained an optimum threshold from several cases. An image whose gray‐scale range has {0,1,…,  *L* − 1} was separated as to destination and background by thresholds *t*. The possibility of gray *i* is *p*_*i*_. The likelihood of objective has *ω*_0_(*t*)=∑_*i*=0_^*t*^*p*_*i*_. The possibility of background is *ω*_1_(*t*)=∑_*i*=*t*+1_^*L*−1^*p*_*i*_. The mean of objective is *u*_0_(*t*)=∑_*i*=0_^*t*^*ip*_*i*_/*ω*_0_. The mean background is *u*_1_(*t*)=∑_*i*=*t*+1_^*L*−1^*ip*_*i*_/*ω*_1_. The formulation of difference between two parts is *d*(*t*)=*ω*_0_(*t*)*ω*_1_(*t*)(*u*_0_(*t*) − *u*_1_(*t*))^2^. An optimum threshold *t*^*∗*^ generates the difference maximal. Therefore, the process of multithreshold segmentation is as follows:

(1) $$\begin{array}{c} d\left(t_{1},t_{2},\ldots ,\;t_{k}\right)=\omega_{0}\omega_{1}{\left(u_{0}-u_{1}\right)}^{2}+\omega_{0}\omega_{2}{\left(u_{0}-u_{2}\right)}^{2}\\ +\omega_{0}\omega_{3}{\left(u_{0}-u_{3}\right)}^{2}\ldots +\omega_{0}\omega_{k}{\left(u_{0}-u_{k}\right)}^{2}\\ +\omega_{1}\omega_{2}{\left(u_{1}-u_{2}\right)}^{2}+\omega_{1}\omega_{3}{\left(u_{1}-u_{3}\right)}^{2}\\ +\ldots +\omega_{1}\omega_{k}\;{\left(u_{1}-u_{k}\right)}^{2}\\ +\ldots +\omega_{k-1}\omega_{k}\;{\left(u_{k-1}-u_{k}\right)}^{2}\\ \omega_{n-1}\left(t\right)=\sum_{i=t_{n-1}+1}^{t_{n}}p_{i},u_{n-1}\left(t\right)=\sum_{i=t_{n-1}+1}^{t_{n}}\frac{ipi}{\omega_{n-1}},\;1\leq n\leq \left(k+1\right). \end{array}$$

Optimum thresholds *t*_1_^*∗*^, *t*_2_^*∗*^,…, *t*_*k*_^*∗*^ create the entire difference maximal as defined below:

(2) $$\begin{array}{c} t_{1}^{*},t_{2}^{*},\ldots ,t_{k}^{*}=Arg\;\max_{0<t_{1}<t_{2}<\ldots <t_{k}}\;d\left(t_{1},t_{2},\ldots ,t_{k}\right).\; \end{array}$$

In this study, the optimal threshold values of the Otsu method are decided by the SOA. The SOA is based on the migration and attacking behavior of the seagulls in nature [18]. The mathematical model of attacking and migrating the prey is described below. The migration (exploration) method inspires how the group of seagulls moves everywhere. In this stage, the seagulls need to fulfill three criteria:

To prevent collision between neighbors (i.e., other seagulls), a further parameter *A* is applied for the assessment of the new search location as follows:

(3) $$\begin{array}{c} {\overset{⟶}{C}}_{s}=A\times {\overset{⟶}{P}}_{s}\left(x\right)\;, \end{array}$$

where ${\overset{⟶}{C}}_{s}$ signifies the location of search agent that does not collide with other searching agents, ${\overset{⟶}{P}}_{s}$ implies the existing location of the search agent, and *x* means the existing iteration as follows:

(4) $$\begin{array}{c} A=f_{c}-\left(x\times \left(\frac{f_{c}}{{\text{Max}}_{\text{iter}\alpha \text{tion}}}\right)\right), \end{array}$$

where *x*=0,  1,  2,   … Max_iteration_.*f*_*c*_ controls the frequency of *A* that is decreased gradually from *f*_*c*_ to 0. In this study, the value of *f*_*c*_ is set to 2. After evading the collision between neighbors, the searching agent is moving towards the direction of the optimal neighbor.

(5) $$\begin{array}{c} {\overset{⟶}{M}}_{s}=B\times \left({\overset{⟶}{P}}_{bs}\left(x\right)-{\overset{⟶}{P}}_{s}\left(x\right)\right). \end{array}$$

Let ${\overset{⟶}{M}}_{s}$ be the position of searching agent ${\overset{⟶}{P}}_{s}$ towards the optimal fit searching agent ${\overset{⟶}{P}}_{bs}$ (viz., appropriate seagull). The behavior of *B* is randomly assigned, that is, accountable for appropriate balancing between exploitation and exploration. *B* is evaluated by

(6) $$\begin{array}{c} B=2\times A^{2}\times r\;d, \end{array}$$

where *r* *d*  represents an arbitrary value within [0.1]. Finally, the searching agent could upgrade its location regarding optimal search agent as follows:

(7) $$\begin{array}{c} {\overset{⟶}{D}}_{s}=\left|{\overset{⟶}{C}}_{s}+{\overset{⟶}{M}}_{s}\right|. \end{array}$$

Let ${\overset{⟶}{D}}_{s}$ be the distance between the optimal fit search agent and search agent (viz., optimal seagulls that fitness value is lesser). The exploitation focuses on exploiting the history and experience of the searching method. Seagulls are capable of changing the speed and angle of attack continuously in migration. They retain their altitude with their weight and wings. During prey attacking, the spiral movement behavior takes place in the air. The *x*, *y*, and *z* planes are shown as follows:

(8) $$\begin{array}{c} x^{\prime }=r\times \;\cos\left(k\right),\\ y^{\prime }=r\times \;\sin\left(k\right),\\ z^{\prime }=r\times k,\\ r=u\times e^{kv}, \end{array}$$

where *r* indicates the radius of every turn of the spiral, *k* represents an arbitrary value within [0 ≤ *k* ≤  2*А*], *u* and *v* denote constant for determining the spiral shape, and *e* represents the base of the natural logarithm. It can be evaluated by

(9) $$\begin{array}{c} {\overset{⟶}{P}}_{s}\left(x\right)=\left({\overset{⟶}{D}}_{s}\times x^{\prime }\times y^{\prime }\times z^{\prime }\right)+{\overset{⟶}{P}}_{bs}\left(x\right), \end{array}$$

where ${\overset{⟶}{P}}_{s}\left(x\right)$ saves the optimal solutions and upgrades the position of another search agent. The presented SOA initiates by an arbitrarily made population. The search agent might update their location regarding the optimum search agent in the iteration method. For smooth transition between exploitation and exploration, *B* is in charge. Therefore, the SOA is regarded as a global optimizer as a result of its good exploitation and exploration capacity.

### 3.3. Feature Extraction

Once the images are segmented, the next stage is to derive a fusion of feature vectors using the CapsNet and EfficientNet models. The two vectors can be defined as follows:

(10) $$\begin{array}{c} f_{\text{CapsNet}1\times n}=\left\{{\text{CapsNet}}_{1\times 1}{\text{,CapsNet}}_{1\times 1}{1\times 2\text{,CapsNet}}_{1\times 11\times 3},\ldots ,{\text{CapsNet}}_{1\times 11\times n}\right\},\\ f_{\text{EfficientNet}\times m}=\left\{{\text{EfficientNet}}_{1\times 1},{\text{EfficientNet}}_{1\times 2},{\text{EfficientNet}}_{1\times 3},\ldots ,{\text{EfficientNet}}_{1\times n}\right\}. \end{array}$$

In addition, the derived individual features are combined into a single vector, using the following equation:

(11) $$\begin{array}{c} \text{Fused}{\left(\text{features vector}\right)}_{1\times q}=\sum_{i=1}^{2}f{\text{CapsNet}}_{1\times n},f{\text{EfficientNet}}_{1\times m}, \end{array}$$

where *f* represents fused vectors (1 × 1186). The entropy is applied on the features vectors to choose optimal features based on the score to the classifier for differentiating the healthier and glioma images.

#### 3.3.1. CapsNet Model

To address the limitations of CNN, Hinton [19] presented a higher dimension vector named “capsule” for representing an entity (object or a portion of object) by a set of neurons instead of an individual neuron. The activity of the neuron in the active capsule signifies different features of a certain entity, that is, existing in an image. Every capsule learns an implicit description of a visual entity that outputs the likelihood and a group of instantiated parameters that includes the accurate posture (orientation, position, and size), albedo, hue, texture, deformation, and so on. The framework of CapsNet is dissimilar to other DL methods. The outcomes of input and output of CapsNet are vector that direction and norm represent the various attributes and existence probability of the entity, correspondingly. The similar levels of capsule assist to forecast the instantiation parameter of a high-level capsule over a conversion matrix, and then dynamic routing is adapted for making the predictions reliable. Once the various predictions are reliable, the high‐level of the single capsule would turn out to be active.

A simple CapsNet framework has been demonstrated in Figure 1, where the framework is shallow by only one fully connected layer (EntityCaps) and two convolution layers (PrimaryCaps and Convl). Especially, Convl is the typical convolution layer that converts the output to PrimaryCaps and images to primary features via a convolutional filter with 13 × 13 × 256  size. In case, the original images are not appropriate for the input of the primary layer of the CapsNet, and the primary feature afterward convolution is adapted. The next convolution layer creates the respective vector as input of the capsule layer. The standard convolutions of all the outputs are a scalar; however, the convolution of PrimaryCaps is dissimilar to the standard one. It is considered as a two-dimensional convolution of eight distinct weights for the input of 15 × 15 × 256. The PrimaryCaps generate a thrity-two size of 11 × 11 steps to 2 convolutions and output. The third layer (EntityCaps) is the output layer, which has nine traditional capsules respective to nine distinct categories.

#### 3.3.2. EfficientNet Model

The EfficientNet technique was utilized as a feature extraction component for generating a helpful group of feature vectors of the input satellite image [20]. The DL is the most well-known framework as DL approaches have been learned significant features in an input image at a different convolutional level similar to the purpose of the human brain. The DL was solving complex problems usually well as well as quickly with high classifier accuracy and lower error rate. The DL approach was contained different modules (convolutional, pooling layer, and fully connected (FC) layers, and activation function). The DL models have the capability of attaining optimal performance over the machine learning models with high computational complexity. Distinct from other existing DL approaches, the EfficientNet structure was a compound scaling manner that employs the compound coefficients to uniformly scale network width, depth, and resolution. An EfficientNet has eight different methods from B0 to B7. The EfficientNet employs inverted bottleneck convolution which is primarily well-known from the MobileNetV2 approach that is a layer that primarily expands the network and next compresses the channel. This structure reduced computation with the factor of 2 as compared with normal convolution, where *f* signifies the filter size. It is depicted that EfficientNetB0 was the easiest of all eight approaches as well as employs minimal parameters. So it can be directly employed EfficientNetB0 to evaluate performance.

#### 3.3.3. DHO-Based Hyperparameter Tuning

In this work, a new metaheuristic DHO method has been developed for the hyperparameter tuning process, stimulated from deer hunting by a group of hunters [21]. For deer hunting, the hunter encircles it as well as gets closer to them by using some strategies. This strategy includes the deliberation of several parameters, such as the deer position, wind angle, and so on. Cooperation between the hunters is another relevant standard that makes hunting very efficient. Lastly, they attain the target as per the location of the successor and leader. The objective function of this presented model is shown below:

(12) $$\begin{array}{c} f\left(x\right)=\;\max\;\left(\text{accuracy}\right). \end{array}$$

The weight optimization with the DHO method is described as follows: because of the unique capabilities of deer, it could escape easily from hunting. The process initiates by a vector of an arbitrary population named hunter. It is described by the following equation:

(13) $$\begin{array}{c} X=\left\{X_{1},X_{2},\;\ldots ,X_{m}\right\}1<j\leq m\;, \end{array}$$

where *m* means the amount of hunter's population (weight), and the overall amount of weight employed to the optimization is denoted as follows. Next, the key parameters such as position angle (weight) and wind angle are employed. The whole searching space is deliberated as a circle; hence, the wind angle can be defined as the circumference of the circle.

(14) $$\begin{array}{c} \theta_{j}=2\pi a, \end{array}$$

where the arbitrary value within = [0,1] is denoted as *a*, and the existing iteration is signified as *J*. Now, *θ* implies the wind angle. Subsequently, the location propagation with the leader position (*X*_*l*_) and successor location (*X*_*s*_) for optimization is presented. The successor location defines the location of subsequent weights, while the leader location defines the primary location of the hunter.

Propagation via (*X*_*l*_). Afterward initiating the optimal location, all the weights in the population try to attain the optimal location. Then, the location updating algorithm starts by modeling the encircling behavior as follows:

(15) $$\begin{array}{c} X_{j+1}=X_{l}-Y\cdot p\cdot \left|L\times X_{l}-X_{j}\right|. \end{array}$$

Let *X*_*j*_ be the location at the existing iteration and the succeeding iteration location is denoted as *X*_*j*+1_. The *Z* and *K* coefficient vectors are involved in this process. The arbitrary value, that is, presented by considering the wind speed is denoted as *p*, and it comprises values *fi*_*i*_*om*0 to 2. The expression to estimate the *Z* and *K* coefficient vectors are given below:

(16) $$\begin{array}{c} Z=\frac{1}{4}\;\log\;\left(j+\frac{1}{j_{\;\max\;}}\right)b,\\ K=2\cdot c, \end{array}$$

where the maximal iteration is denoted as *j*_ max _. The *b* variable has values ranging from −1 to 1, besides the value of other variables lies within [0,1]. The first location of the hunter is signified as (*X*,  *Y*) that gets upgraded according to the location of prey. Both *Z* and *K* coefficient vectors are modified to reach the optimal location (*X*_*b*_,  *Y*_*b*_). When the value of *p*<1, the location updation algorithm takes place that implies the hunter could arbitrarily move in a different direction without considering the angle location. *Propagation through Angle Location*. The angle location updating is considered to rise the searching space. For making the hunting method more efficient, it is crucial to describe the angle location of the hunter. It can be implemented by

(17) $$\begin{array}{c} X_{j+1}=X_{l}-p\cdot \left|\;\cos\;\left(v\right)\times X_{l}-X_{j}\right|, \end{array}$$

where p denotes the arbitray values and the optimal location can be depicted as *B*=*φ*_*j*+1_, *X*_*b*_*j*__ and *p*. The individual location is found the opposite to the angle location; hence, the prey does not have any alertness of the hunter. *Propagation via Successor Location*. In the exploration, the vector *K*  is presented within the encircle behavior. At first, the arbitrary searching method is performed by considering the *K* values as less than 1. Lastly, the location updating algorithm takes place based on a successor location instead of considering the optimal location. Next, the global searching is carried out by

(18) $$\begin{array}{c} X_{j+1}=X_{s}-Z\cdot p\cdot \left|K\times X_{s}-X_{j}\right|. \end{array}$$

The location updating method is performed for identifying the optimal location (viz., termination condition).

### 3.4. Image Classification

At the final stage, the FSVM model is applied to determine the suitable class labels for the test images. In conventional SVM, each data point is regarded as equally significant and allotted a similar penal variable. Though in several real-time classification applications, few sample points, such as noises/outliers, may not be accurately allotted to one of these two classes, and all the sample points do not have a similar meaning to the decision surface. The hyperplanes in the SVM model are shown in Figure 2. To resolve this issue, the FSVM concept was initially presented [22]. Fuzzy membership to all the sample points is proposed so that discrete sample points might generate distinct contributions to the generation of decision surfaces. The trained sample is considered as follows:

(19) $$\begin{array}{c} S=\left\{\left(x_{i},y_{i},s_{i}\right),\;i=1,\ldots ,\;N\right\}. \end{array}$$

Let *x*_*i*_ ∈ *R*^*n*^ be the *n*‐dimensional sample point, *y*_*i*_ ∈ {−1, +1} signifies its class label, and *s*_*i*_(*i*=1,…, *N*) implies a fuzzy membership that fulfills *σ* ≤ *s*_i_ ≤ 1 with small constant *σ* > 0. The quadratic optimization problems for classification can be represented by

(20) $$\begin{array}{c} \underset{w,s,\xi }{\min}\frac{1}{2}w^{T}w+C\sum_{i‐1}^{l}s_{i}\xi_{i},\\ s.t.\;y_{i}\left(w^{T}x_{i}+b\right)\geq 1-\xi_{i},\;\xi_{i}\geq 0,\;i=1,\ldots ,\;l, \end{array}$$

where *w* indicates a standard vector of the separating hyperplane, *b* denotes a bias, and *C* represents a parameter that needs to be determined earlier to control the trade-offs amongst the cost of misclassification error and the classification margin. As *s*_*i*_ represent the attitude of the respective point *x*_*i*_ towards one class and the slack parameter *ξ*_*i*_ is a measure of error, the *s*_*i*_*ξ*_*i*_ the term could consider the measure of error with discrete weights. It is considered that the larger the *s*_*i*_ is, the more significantly the respective point is treated; the lower the *s*_*i*_ is, the less outstandingly the respective point is treated. Hereafter, FSVM could discover a strong hyperplane by maximalizing the margin by letting some misclassification of lesser significant points.

For resolving the FSM problems, (2) is transformed into the subsequent dual problem by introducing Lagrangian multiplier *α*_*i*_ as follows:

(21) $$\begin{array}{c} \underset{\alpha }{\max}\sum_{i=1}^{N}\alpha_{i}-\frac{1}{2}\sum_{i=1}^{N}\sum_{j=1}^{N}\left.\alpha_{i}\alpha_{j}y_{i}y_{j}x_{i}x_{j}\right),\\ s.t.\sum_{i=1}^{N}y_{i}\alpha_{i}=0,\;0\leq \alpha_{i}\leq s_{i}\;C,\;i=1,\ldots ,N. \end{array}$$

When compared to the typical SVM, the above stated has only a small difference, that is, the upper bounds of the value of *α*_*i*_. By solving this dual problem in (3) for optimal *α*_*i*_, *w*, and *b* could be recovered in the same way as in the typical SVM.

## 4. Performance Validation

The performance validation of the proposed model takes place using a benchmark CT ICH data set, including 341 images [23]. It comprises 171 images under epidural (EPI) class, 24 images under intraventricular (IVT), 72 images under intraparenchymal (IPC), 56 images under subdural (SBD), and 18 images under subarachnoid (SAD) class. The size of the image is 512 ∗ 512 pixels.  Figure 3 shows the sample test images. The data sets include ICH masks and CT scans, in JPG and NIfTI format at PhysioNet repository. NIfTI is a type of file format for neuroimaging, which is used very commonly in imaging informatics for neuroscience and even neuroradiology research.

Figure 4 showcases the confusion matrix of the AICH-FDLSI technique on the test images under run-1. The figure reported that the AICH-FDLSI technique has classified 19 images under IVT, 64 images under IPC, 12 images under SAD, 170 images under EPI, and 54 images under SBD.

Table 1 reports the ICH classification results analysis of the AICH-FDLSI technique under run-1. The results demonstrated that the AICH-FDLSI technique has classified the IVT class with the sens_*y*_, spec_*y*_, prec_*n*_,   and accu_*y*_ of 0.7917, 0.9811, 0.7600, and 0.9677, respectively. In line with, the AICH-FDLSI technique has identified the IPC class with the sens_*y*_, spec_*y*_, prec_*n*_, and accu_*y*_ of 0.8889, 0.9888, 0.9552, and 0.9677, respectively. Moreover, the AICH-FDLSI technique has identified the instances under SBD with the sens_*y*_, spec_*y*_, prec_*n*_, and accu_*y*_ of 0.9643, 0.9895, 0.9474, and 0.9853, respectively.

Figure 5 displays the confusion matrix of the AICH-FDLSI technique on the test images under run-2. The figure revealed that the AICH-FDLSI technique has identified 20 images under IVT, 64 images under IPC, 12 images under SAD, 170 images under EPI, and 54 images under SBD.

Table 2 offers the ICH classification results analysis of the AICH-FDLSI technique under run-2. The experimental values stated that the AICH-FDLSI technique has classified the IVT class with the sens_*y*_, spec_*y*_, prec_*n*_, and accu_*y*_ of 0.8333, 0.9811, 0.7692, and 0.9707, respectively. Moreover, the AICH-FDLSI technique has categorized the IPC class with the sens_*y*_, spec_*y*_, prec_*n*_, and accu_*y*_ of 0.8889, 0.9888, 0.9552, and 0.9677, respectively. Eventually, the AICH-FDLSI technique has determined the images under SBD with the sens_*y*_, spec_*y*_, prec_*n*_, and accu_*y*_ of 0.9643, 1.0000, 1.0000, and 0.9941, respectively.

Figure 6 demonstrates the confusion matrix of the AICH-FDLSI technique on the test images under run-3. The figure shows that the AICH-FDLSI technique has identified 22 images under IVT, 64 images under IPC, 12 images under SAD, 170 images under EPI, and 54 images under SBD.  Table 3 depicts the ICH detection performance analysis of the AICH-FDLSI technique under run-1. The results show that the AICH-FDLSI technique has effectively identified the IVT class with the sens_*y*_, spec_*y*_, prec_*n*_, and accu_*y*_ of 0.9167, 0.9811, 0.7857, and 0.9765, respectively. Meanwhile, the AICH-FDLSI technique has identified the IPC class with the sens_*y*_, spec_*y*_, prec_*n*_, and accu_*y*_ of 0.8889, 0.9888, 0.9552, and 0.9677, respectively. Lastly, the AICH-FDLSI technique has identified the instances under SBD with the sens_*y*_, spec_*y*_, prec_*n*_, and accu_*y*_ of 0.9643, 1.0000, 1.0000, and 0.9941, respectively.

Table 4 and Figure 7 offer an overall result analysis of the AICH-FDLSI technique under three different runs. The results show that the AICH-FDLSI technique has accomplished maximum classification performance under three test runs. For instance, under run-1, the AICH-FDLSI technique has classified the ICH with the sens_*y*_, spec_*y*_, prec_*n*_, and accu_*y*_ of 0.8611, 0.9812, 0.8950, and 0.9742, respectively. Likewise, under run-2, the AICH-FDLSI technique has classified the ICH with the sens_*y*_, spec_*y*_, prec_*n*_, and accu_*y*_ of 0.8695, 0.9810, 0.9052, and 0.9754, respectively. Similarly, under run-3, the AICH-FDLSI technique has classified the ICH with the  sens_*y*_, spec_*y*_, prec_*n*_, and accu_*y*_ of 0.8861, 0.9833, 0.9106, and 0.9777, respectively.

Figure 8 investigates the accuracy graph of the AICH-FDLSI technique on the test data set. The figure demonstrated that the AICH-FDLSI technique has resulted in improved training and validation accuracies.

The loss graph analysis of the AICH-FDLSI technique takes place on the test data set in Figure 9. The results highlighted that the loss values tend to decrease with the increased epoch count, and it is observable that the validation loss seems to be lower than the training loss.

Table 5 provides a brief result analysis of the AICH-FDLSI with recent techniques. A brief sens_*y*_ analysis of the AICH-FDLSI technique with existing approaches [16,24–27] is provided in Figure 10. The figure shows that the UNet, WANN, and SVM techniques have attained lower sens_*y*_ values of 63.10%, 60.18%, and 76.38%, respectively. Eventually, the WEM-DCNN and convolutional NN techniques have resulted in reasonable sens_*y*_ of 83.33%, and 87.06%, respectively. But the AICH-FDLSI technique has surpassed the other ones with the increased sens_*y*_ of 88.61%.

A comparative prec_*n*_ analysis of the AICH-FDLSI technique with other techniques is shown in Figure 11. The figure reported that the WANN and SVM techniques have attained lower prec_*n*_ values of 70.08% and 77.53%, respectively. Along with that, the UNet, WEM-DCNN, and convolutional NN techniques have obtained moderate prec_*n*_ of 88.19%, 89.90%, and 87.98%, respectively. However, the AICH-FDLSI technique has outperformed the other ones with the higher prec_*n*_ of 91.06%.

Table 6 offers a comparative results analysis of the AICH-FDLSI with recent techniques in terms of spec_*y*_ and accu_*y*_.  Figure 12 depicts the comparative spec_*y*_ analysis of the AICH-FDLSI system with other techniques. From the figure, it is notable that the UNet, WANN, Res-NexT, convolutional NN, and SVM techniques have accomplished minimal classification performance with the spec_*y*_ values of 88.60%, 70.13%, 90.42%, 88.18%, and 77.53%, respectively. Next to that, the DN-ELM and WEM-DCNN techniques have resulted to reasonable spec_*y*_ of 97.70%, and 97.48%, respectively. However, the AICH-FDLSI technique has gained improved performance with the superior spec_*y*_ of 98.33%.

Figure 13 portrays the comparative accu_*y*_ analysis of the AICH-FDLSI system with other techniques. From the figure, it is notable that the UNet, WANN, Res-NexT, convolutional NN, WEM-DCNN, and SVM techniques have accomplished minimal classification performance with the accu_*y*_ values of 87%, 69.78%, 89.30%, 87.56%, 88.35%, and 77.32%, respectively. Following that, the DN-ELM model has offered competitive accu_*y*_ of 96.34%. But the AICH-FDLSI technique has surpassed the other ones with the maximum accu_*y*_ of 97.77%.

Finally, the CT analysis of the AICH-FDLSI methodology with recent approaches is shown in Figure 14. The results portrayed that the WANN, Res-NexT, and SVM models have obtained worse outcomes with maximum CT of 78 s, 80 s, and 89 s, respectively. Following that, the WEM-DCNN and convolutional NN techniques have attained moderately closer CT of 75% and 74%, respectively. Along with that, the DN-ELM and UNet models have obtained reasonable CT of 29 s and 42 s, respectively. However, the AICH-FDLSI technique has accomplished improved performance with the CT of 24 s. From the above-mentioned results, it is evident that the AICH-FDLSI process is found to be an efficient tool for ICH detection and classification.

## 5. Conclusion

This paper has developed a novel AICH-FDLSI technique for ICH detection and classification. The proposed AICH-FDLSI technique encompasses MF-based preprocessing, SOA with Otsu multilevel thresholding-based segmentation, fusion-based feature extraction, DHO-based feature extraction, and FSVM-based classification. The application of SOA and DHO algorithms helps improvise the overall ICH classification performance. To showcase the improved classifier results of the proposed model, a wide range of experiments is performed using the test benchmark intracranial haemorrhage data set. The experimental outcome stated that the AICH-FDLSI model has reached a proficient performance. Therefore, the proposed AICH-FDLSI technique can be applied as a proficient tool for ICH diagnosis and classification. In the future, the ICH classification performance of the AICH-FDLSI technique can be improvised by the use of hybrid DL models.

## Figures and Tables

**Figure 1:** Process of CapsNet [19].

**Figure 2:** SVM hyperplanes.

**Figure 3:** Sample images.

**Figure 4:** Confusion matrix of AICH-FDLSI technique under run-1.

**Figure 5:** Confusion matrix of AICH-FDLSI technique under run-2.

**Figure 6:** Confusion matrix of AICH-FDLSI technique under run-3.

**Figure 7:** Results analysis of AICH-FDLSI technique under three different runs.

**Figure 8:** Accuracy graph analysis of AICH-FDLSI technique.

**Figure 9:** Loss graph analysis of AICH-FDLSI technique.

**Figure 10:** Comparative sens_*y*_ analysis of AICH-FDLSI technique.

**Figure 11:** Comparative prec_*n*_ analysis of AICH-FDLSI technique.

**Figure 12:** Comparative spec_*y*_ analysis of AICH-FDLSI technique.

**Figure 13:** Comparative accu_*y*_ analysis of AICH-FDLSI technique.

**Figure 14:** Comparative CT analysis of AICH-FDLSI technique.

**Table 1:** ICH classification results analysis of AICH-FDLSI technique on test run-1.

Classes	Sensitivity	Specificity	Precision	Accuracy
IVT	0.7917	0.9811	0.7600	0.9677
IPC	0.8889	0.9888	0.9552	0.9677
SAD	0.6667	0.9938	0.8571	0.9765
EPI	0.9942	0.9529	0.9551	0.9736
SBD	0.9643	0.9895	0.9474	0.9853
Average	0.8611	0.9812	0.8950	0.9742

**Table 2:** ICH classification results analysis of AICH-FDLSI technique on test run-2.

Classes	Sensitivity	Specificity	Precision	Accuracy
IVT	0.8333	0.9811	0.7692	0.9707
IPC	0.8889	0.9888	0.9552	0.9677
SAD	0.6667	0.9938	0.8571	0.9765
EPI	0.9942	0.9412	0.9444	0.9677
SBD	0.9643	1.0000	1.0000	0.9941
Average	0.8695	0.9810	0.9052	0.9754

**Table 3:** ICH classification results analysis of AICH-FDLSI technique on test run-3.

Classes	Sensitivity	Specificity	Precision	Accuracy
IVT	0.9167	0.9811	0.7857	0.9765
IPC	0.8889	0.9888	0.9552	0.9677
SAD	0.6667	0.9938	0.8571	0.9765
EPI	0.9942	0.9529	0.9551	0.9736
SBD	0.9643	1.0000	1.0000	0.9941
Average	0.8861	0.9833	0.9106	0.9777

**Table 4:** Overall ICH results analysis of AICH-FDLSI technique.

No. of runs	Sensitivity	Specificity	Precision	Accuracy
Run-1	0.8611	0.9812	0.8950	0.9742
Run-2	0.8695	0.9810	0.9052	0.9754
Run-3	0.8861	0.9833	0.9106	0.9777

**Table 5:** Comparative results analysis of AICH-FDLSI with recent methods-I.

Methods	Sensitivity	Precision
AICH-FDLSI	88.61	91.06
UNet model	63.10	88.19
WANN	60.18	70.08
WEM-DCNN	83.33	89.90
Convolutional NN	87.06	87.98
SVM	76.38	77.53

**Table 6:** Comparative results analysis of AICH-FDLSI with recent methods-II.

Methods	Specificity	Accuracy
AICH-FDLSI	98.33	97.77
DN-ELM	97.70	96.34
UNet model	88.60	87.00
WANN	70.13	69.78
Res-NexT	90.42	89.30
WEM-DCNN	97.48	88.35
Convolutional NN	88.18	87.56
SVM	79.41	77.32

## Data Availability

The data set used in this paper is publicly available at https://physionet.org/content/ct-ich/1.3.1/

## References

[1] Majumdar A., Brattain L., Telfer B., Farris C., Scalera J. Detecting intracranial hemorrhage with deep learning.

[2] Arbabshirani M. R., Fornwalt B. K., Mongelluzzo G. J. (2018). Advanced machine learning in action: identification of intracranial hemorrhage on computed tomography scans of the head with clinical workflow integration. *NPJ digital medicine*.

[3] Gou X., He X. (2021). Deep learning-based detection and diagnosis of subarachnoid hemorrhage. *Journal of Healthcare Engineering*.

[4] Kumar N., Narayan Das N., Gupta D., Gupta K., Bindra J. (2021). Efficient automated disease diagnosis using machine learning models. *Journal of Healthcare Engineering*.

[5] Luo L., Xu X., Jiang Y., Zhu W. (2019). Predicting intracerebral hemorrhage patients’ length-of-stay probability distribution based on demographic, clinical, admission diagnosis, and surgery information. *Journal of healthcare engineering*.

[6] Chen H., Khan S., Kou B., Nazir S., Liu W., Hussain A. (2020). A Smart Machine Learning Model for the Detection of Brain Hemorrhage Diagnosis Based Internet of Things in Smart Cities. *Complexity*.

[7] Ginat D. T. (2020). Analysis of head CT scans flagged by deep learning software for acute intracranial hemorrhage. *Neuroradiology*.

[8] Mansour R. F., Aljehane N. O. (2021). An optimal segmentation with deep learning based inception network model for intracranial hemorrhage diagnosis. *Neural Computing & Applications*.

[9] Anupama C. S. S., Sivaram M., Lydia E. L., Gupta D., Shankar K. (2020). Synergic Deep Learning Model–Based Automated Detection and Classification of Brain Intracranial Hemorrhage Images in Wearable Networks. *Personal and Ubiquitous Computing*.

[10] Venugopal D., Jayasankar T., Yacin Sikkandar M. (2021). A novel deep neural network for intracranial haemorrhage detection and classification. *Computers, Materials & Continua*.

[11] Lee J. Y., Kim J. S., Kim T. Y., Kim Y. S. (2020). Detection and classification of intracranial haemorrhage on CT images using a novel deep-learning algorithm. *Scientific Reports*.

[12] Wang T., Song N., Liu L. (2021). Efficiency of a deep learning-based artificial intelligence diagnostic system in spontaneous intracerebral hemorrhage volume measurement. *BMC Medical Imaging*.

[13] Yu N., Yu H., Li H., Ma N., Hu C., Wang J. (2021). A Robust Deep Learning Segmentation Method for Hematoma Volumetric Detection in Intracerebral Hemorrhage. *Stroke*.

[14] Luong K. G., Duong H. N., Van C. M. A computer-aided detection to intracranial hemorrhage by using deep learning: a case study.

[15] Ngo D. T., Nguyen D. B., Nguyen H. T., Pham H. H., Nguyen H. Q. (2020).

[16] Hssayeni M. D., Croock M. S., Salman A. D., Al-khafaji H. F., Yahya Z. A., Ghoraani B. (2020). Intracranial hemorrhage segmentation using a deep convolutional model. *Data*.

[17] Akagic A., Buza E., Omanovic S., Karabegovic A. May. Pavement crack detection using Otsu thresholding for image segmentation.

[18] Dhiman G., Kumar V. (2019). Seagull optimization algorithm: theory and its applications for large-scale industrial engineering problems. *Knowledge-Based Systems*.

[19] Sabour S., Frosst N., Hinton G. E. (2017). Dynamic Routing between Capsules. https://arxiv.org/abs/1710.09829.

[20] Marques G., Agarwal D., de la Torre Díez I. (2020). Automated medical diagnosis of COVID-19 through EfficientNet convolutional neural network. *Applied Soft Computing*.

[21] Brammya G., Praveena S., Ninu Preetha N. S., Ramya R., Rajakumar B. R., Binu D. (2019). Deer hunting optimization algorithm: a new nature-inspired meta-heuristic paradigm. *The Computer Journal*.

[22] Fan Q., Wang Z., Li D., Gao D., Zha H. (2017). Entropy-based fuzzy support vector machine for imbalanced datasets. *Knowledge-Based Systems*.

[23] Hssayeni M. D., Croock M. S., Salman A. D., Al-khafaji H. F., Yahya Z. A., Ghoraani B. (2020). Computed Tomography Images for Intracranial Hemorrhage Detection and Segmentation. *Intracranial Hemorrhage Segmentation Using A Deep Convolutional Model. Data*.

[24] Santhoshkumar S., Varadarajan V., Gavaskar S., Amalraj J. J., Sumathi A. (2021). Machine learning model for intracranial hemorrhage diagnosis and classification. *Electronics*.

[25] Davis V., Devane S. Diagnosis & classification of brain hemorrhage.

[26] Danilov G., Kotik K., Negreeva A. (2020). Classification of intracranial hemorrhage subtypes using deep learning on CT scans. *Studies in Health Technology and Informatics*.

[27] Karki M., Cho J., Lee E. (2020). CT window trainable neural network for improving intracranial hemorrhage detection by combining multiple settings. *Artificial Intelligence in Medicine*.

